# Qi Sui Zhu Shui Plaster Inhibits AQP1 and MAPK Signaling Reduces Liver Damage Induced by Cirrhotic Ascites

**DOI:** 10.1155/2022/9928546

**Published:** 2022-03-30

**Authors:** Rong Zhen Zhang, Yin Liu, Min Li, Yong Lin Huang, Zhen Heng Song

**Affiliations:** ^1^Department of Hepatology, The First Affiliated Hospital of Guangxi University of Chinese Medicine, Nanning, China; ^2^Department of Medical Laboratory, The First Affiliated Hospital of Guangxi University of Chinese Medicine, Nanning, China; ^3^Department of Hepatology, Guangxi University of Chinese Medicine, Nanning, China

## Abstract

**Objective:**

At present, there is no special treatment for cirrhotic ascites in modern medicine. Qi Sui Zhu Shui plaster (QSZSP) has been used in ascites. The purpose of this study was to investigate the mechanism of action of QSZSP in the treatment of cirrhotic ascites and its relationship with aquaporin 1 (AQP1).

**Methods:**

Twenty-four rats were divided into four groups, six rats in each group. Carbon tetrachloride-olive oil is injected into modeling. The control and model groups are treated with blank gel plaster (2 cm × 2 cm), QSZSP low-dose group is treated with Qi Sui Zhu Shui plaster (1 cm × 1 cm), and QSZSP high-dose group is treated with Qi Sui Zhu Shui plaster (2 cm × 2 cm). The changes in body weight and abdominal circumference were measured, the histopathological changes in liver, kidney, and peritoneum were observed in HE staining, the biochemical indexes related to liver function were detected, and the changes in AQP1 expression and the activation of MAPK pathway in the liver, kidney, and peritoneal tissues were evaluated in IHC staining and Western blot.

**Results:**

After one week of injection of carbon tetrachloride-olive oil, the rats in the model group increased their body weight slowly, the abdominal circumference of the model rats continued to increase with time. After 16 weeks of construction of the cirrhotic ascites model, the liver, kidney, and peritoneum were significantly damaged, and the serum levels of TBiL, AST, ALT, Cr, BUN, K, Na, and Ca in the rats were significantly higher (*P* < 0.001) and ALB levels were significantly lower (*P* < 0.001) than those in the control group. After 4 weeks of treatment, the liver, kidney, and peritoneal injury were improved. TBiL, AST, ALT, Cr, BUN, K, Na, and Ca levels were significantly lower (*P* < 0.001) and ALB levels were significantly higher (*P* < 0.001) than those in the model group. The protein expression of AQP1, p-ERK, p-JNK, and p-p38 was found to be inhibited in the liver, kidney, and peritoneum.

**Conclusion:**

QSZSP inhibits the protein expression of AQP1 and MAPK signaling pathway in the liver, peritoneum, and kidney to alleviate liver, kidney, and peritoneal injury caused by cirrhotic ascites, thus reducing the abnormal growth of abdominal circumference.

## 1. Introduction

Cirrhosis is a common clinical disease, which is caused by a series of pathological changes such as degeneration, necrosis, regeneration, and fibrous tissue proliferation of hepatocytes due to the persistent or repeated action of various pathogenic factors on the liver tissues, mainly manifesting as liver function decline [1]. The worldwide prevalence of cirrhosis is unknown. The prevalence of cirrhosis in the United States is about 0.15%–0.27% [2]. 69% of people do not know they have cirrhosis, and diabetes, alcohol abuse, hepatitis C and hepatitis B, being male, and being older are all associated with cirrhosis [3]. Regardless of the etiology, 50% of patients with cirrhosis will develop cirrhotic cardiomyopathy [4]. The 2017 National Vital Statistics Report for the United States reported that approximately 4.5 million adults, or 1.8% of the adult population, have chronic liver disease and cirrhosis. 41,473 people died from chronic liver disease and cirrhosis [5].

Ascites is the most prominent clinical manifestation of cirrhosis. It is the abnormal fluid accumulation in the abdominal cavity. About 60% of patients with compensatory cirrhosis develop abnormal peritoneal fluid accumulation within 10 years of diagnosis high incidence and poor prognosis of cirrhotic ascites, especially refractory ascites, can induce many fatal complications, which seriously affect the quality of life and survival rate of cirrhotic patients [7]. 90% of liver cancer cases are associated with the presence of cirrhosis [8].

Traditional Chinese medicine (TCM) has the effect of blocking or delaying malignancy and has low toxicity [9]. Long-term use of Chinese herbs can reduce the risk of cirrhosis in patients with chronic hepatitis B [10]. Qi Sui Zhu Shui plaster (QSZSP) consists of *Radix Astragali*, *Radix Kansui*, *Radix Aucklandiae*, *Poria*, *Herba Leonuri*, *Radix Salviae miltiorrhizae*, and *Pericarpium Arecae*. A previous clinical study found that QSZSP adjuvant treatment of patients with cirrhotic ascites resulted in improved urine output, 24 h urinary sodium excretion, reduced creatinine and total bilirubin levels, increased albumin content, and improved ascites recurrence rate after 3 months of continuous treatment with QSZSP [11]. There are few studies on QSZSP and cirrhotic ascites. In the history of research on the components in QSZSP and cirrhosis of the liver, Xiaozhang Tie as an adjuvant to primary therapy of cirrhotic ascites is safe [12]. Salviae miltiorrhizae significantly ameliorates cirrhosis and portal hypertension [13]. Further studies are needed on the agents of action of QSZSP in the treatment of cirrhotic ascites.

In 1991, CHIP28 was shown to function as a water channel, and subsequently, CHIP28 was renamed aquaporins [14, 15]. Thirteen aquaporins (AQP0-AQP12) have been identified [16–18]. Aquaporins have three isoforms. The first subtype transports only water molecules, the second subtype transports water molecules, urea, glycerol, etc., and the third subtype transports channels continuously open, without energy consumption or regulation [19–21]. Aquaporin 1 (AQP1) belongs to the first subtype, which exists as a tetramer and allows only water molecules to be transported across the membrane, and it is an independent water channel [22, 23]. The liver, peritoneum, and kidney are the organs in close contact, and AQP1 happens to be distributed in the liver, peritoneum, and kidney [24]. The water content of the human body is 70% of body weight, and abnormal water production-absorption-excretion in the peritoneal cavity is a key factor in the formation of ascites [19]. AQP1 is one of the aquaporins involved only in the transport of water molecules. Ascites in cirrhosis leads to increased accumulation of fluid in the liver, and the excess fluid is transferred to the peritoneum, which does not reabsorb enough water and eventually leads to increased reabsorption of water by the kidney, so AQP1 may be an important intermediate to study the metabolism of ascites.

Initially, cirrhosis leads to decreased liver function and increased fluid accumulation in the abdominal and thoracic cavities, forming ascites [25]. Ascites occurs commonly in cirrhosis [6]. Ascites is the abnormal fluid accumulation in the abdominal cavity [6]. Cirrhotic ascites can lead to kidney dysfunction [26]. In peripheral arterial vasodilation hypothesis, the kidney is involved in all 5 stages of ascites [27]. By linking AQP1 expression in the liver, peritoneum, and kidney, we propose a “liver-peritoneal-kidney” axis in cirrhotic ascites and suggest that it plays a critical role in the formation of cirrhotic ascites. It has been reported that AQP1 is regulated by MEK1/2 inhibitors in glial cells [28]. In prostate cancer cells, AQP1 protein expression levels are regulated by p38MAPK [29]. In human pleural mesothelial cells, peptidoglycan inhibits p38 MAPK regulation of AQP1 protein expression [30]. Therefore, the MAPK pathway would be a direction of AQP1 changes in the “liver-peritoneal-kidney” axis.

The role of QSZSP in the treatment of cirrhotic ascites and its relationship with AQP1 has not been reported yet. We speculate that the “liver-peritoneal-kidney” axis is a functional axis of water metabolism with aquaporins as the common material basis, which is involved in the “production-absorption-excision” of peritoneal fluid and plays a key role in the formation of cirrhotic ascites. The MAPK pathway may mediate QSZSP regulation of AQP1. Therefore, in this study, we treated rats with cirrhotic ascites *in vitro* with QSZSP, observed the histopathological changes in liver, kidney, and peritoneum, and evaluated the changes in AQP1 expression and activation of MAPK pathway in the liver, kidney, and peritoneal tissues to elucidate the effect of QSZSP in treating cirrhotic ascites and its mechanism.

## 2. Material and Methods

### 2.1. Regents

The reagents used are as follows: carbon tetrachloride (C805332) from Macklin, olive oil from Yihai Kerry Golden Dragon Fish Cereals, Oils and Foodstuffs Co., Ltd. (China), xylene and absolute ethanol from National Pharmaceutical Group Chemical Reagent Co., Ltd. (China), eosin (E8090) and neutral resin (G8590) from Solarbio (China), and hematoxylin (G1004) from Servicebio.

### 2.2. Qi Sui Zhu Shui Plaster Process

Qi Sui Zhu Shui plaster consists of Radix Astragali, Radix Kansui, Radix Aucklandiae, Poria, Herba Leonuri, Radix Salviae miltiorrhizae, and Pericarpium Arecae. The above seven Chinese medicines were purchased from the First Affiliated Hospital of Guangxi University of Traditional Chinese Medicine, in accordance with the provisions of the “Chinese Pharmacopoeia” 2010 edition.

12 ml of water is added to each 1 g of Radix Astragali, Poria, and Herba Leonuri and soaked for 30 min, water reflux extraction is repeated 3 times, 1.5 h each time, and the extracts are combined and filtered. 6 ml of 85% ethanol is added to each 1 g of Radix Kansui, Radix Aucklandiae, Radix Salviae miltiorrhizae, and Pericarpium Arecae and soaked for 30 min, water reflux extraction is repeated twice, 1.5 h each time, and the extracts are combined and filtered. The above two extracts were combined and dried under a vacuum to prepare dry powder. The base consists of 60% SodiuM acrylate, 30% carbomer, 10% Aluminium glycinate, and 6 times Glycerine. The penetration enhancer consists of 50% Azone and 50% propylene glycol. The base, penetration enhancer, and dry powder are mixed. Coater (RK-200, Tianjin Ruikang Babu Pharmaceutical Biotechnology Co., Ltd.) producing QSZSP is used. The hydrogel paste is prepared by RK-200 hydrogel coating machine (Tianjin Ruikang Babu Pharmaceutical Biotechnology Co.). Each tablet of this product contains Astragalus methyloside (C_41_H_68_O_14_) in Radix Astragali, not less than 0.6932 mg, and Euphorbia grandis dienol (C_30_H_50_O) in Radix Kansui, not less than 1.4766 mg.

### 2.3. Animal

Animals from three Gorges University, twenty-four rats, male, weighing 200∼250 g, were raised under the condition of no specific pathogen (specific pathogen free, SPF). The feeding environment is 22–26°C, 50%–60% of relative humidity. Modeling will begin in two weeks. Carbon tetrachloride-olive oil in 4 : 6 proportion, intraperitoneal injection dose of 3 mL/kg body weight, and injections were given twice a week (the four days and the seven days) for eleven weeks. For the control group, isotonic intraperitoneal injection of an equal amount of olive oil was given. The weight and abdominal circumference are measured before each injection. During the period, distilled water with 75% medical alcohol was used to prepare 10% concentration of drinking water for rats. Finally, four weeks of treatment, the body weight (Table 1), and abdominal circumference (Table 2) of the rats were measured twice a week for 15 weeks.

### 2.4. Treating and Sampling

Twenty-four rats were divided into four groups, six rats in each group, all rats were dehaired on the abdomen, and the dehairing area was 3 cm × 3 cm. Control group (Con) is treated with blank gel plaster (2 cm × 2 cm); model group (Mod), blank gel plaster (2 cm × 2 cm); QSZSP low-dose group, Qi Sui Zhu Shui plaster (1 cm × 1 cm); and QSZSP high-dose group, Qi Sui Zhu Shui plaster (2 cm × 2 cm). These were applied to the abdominal skin of depilated rats once a day for 6 h for 4 weeks. Carbon tetrachloride-olive oil was injected subcutaneously into the back once a week during treatment to prevent reversal of cirrhosis. After four weeks, the animals were killed by anesthesia and bloodletting. If the animals were not dead, the animals were anesthetized to death with pentobarbital sodium overdose (100 mg/kg). After anesthesia, the animals died without breathing or heartbeat. The filter paper method is used to obtain ascites. The blood from the abdominal aorta is collected and centrifuged, and serum is collected. An appropriate amount of liver tissue, kidney tissue, and peritoneal tissue is cut and fixed with 4% paraformaldehyde. In addition, the tissues of liver, peritoneum, and kidney were stored in an ultra-low-temperature refrigerator at −80°C. The fixed liver, kidney, and peritoneal tissues of rats were dehydrated and embedded in wax. The sections were frozen at −20°C and cut into a thickness of 3 *μ*m, a water bath was used to stretch the sections, the sections were attached to slides, and the sections were stored at 4°C for backup.

### 2.5. Hematoxylin and Eosin (HE) Staining

The sections were stained in hematoxylin solution for 4 min, followed by rinsing with running tap water for 2 min and 15 s. The sections were then counterstained with eosin solution for 3 min. Cleaning was carried out at 80% and 95% ethanol, respectively, for 30 s each. The sections were then cleared in xylene for 3 s and mounted with neutral balsam. After staining, the sections were observed using a microscope, and Leica Application Suite was used to collect and analyze the relevant parts of the samples.

### 2.6. Biochemical Analysis

After the serum samples were thawed at 4°C, the serum samples were detected by Shenzhen Mindray BS420 Automatic Biochemical Analyzer, and TBiL, AST, ALT, ALB, Cr, BUN, K, Na, and Ca concentrations were determined with the Shenzhen Mairui (Shenzhen, China) Matching Biochemical Kit.

### 2.7. Immunohistochemical Staining

The protein expression of AQP1 in the liver, peritoneum, and kidney tissues was examined by immunohistochemistry. The slides were baked at 65°C for 1 h, soaked in xylene for 30 min, and hydrated in gradient alcohol. 1 mM Tris-EDTA buffer solution (G1203, Servicebio) was used for 18 min repair at 125°C and 103 kPa, incubated with 3% H_2_O_2_ (National Pharmaceutical Group Chemical Reagent Co., Ltd., China) for 10 min, incubated with 10% goat serum (SL038, Solarbio) for 30 min, and titrated with primary antibody AQP1 (PAB45863, Bioswamp), peritoneum dilution 1 : 250, and liver and kidney dilution 1 : 400 at 4°C overnight. The sections were transferred from 4°C to room temperature and left for 45 min. Treated with Max Vision TM HRP-Polymer anti-Rabbit secondary antibody (KIT-5020, MXB) for 60 min at 37°C. Treated with DAB (DA1010, Solarbio) until the sections change color. Soak the sections in turn, hematoxylin 3 min, 75% alcohol 5 min, 85% alcohol 5 min, 95% alcohol 5 min, 100% alcohol 10 min, xylene 10 min. Neutral resins seal sections. Leica Application Suite image system was used to capture the relevant parts of the sample. The nuclei were stained blue with hematoxylin, and the DAB showed positive brownish yellow.

### 2.8. Western Blot

The protein levels of p38, p-p38, ERK1/2, p-ERK1/2, JNK1/2/3, p-JNK1/2/3, and AQP1 in the liver, peritoneum, and kidney tissues were analyzed by Western blot. Tissue samples were homogenized in RIPA lysate (R0010, Solarbio) containing protease inhibitor at 4°C and centrifuged at 12000 g for 15 min. The concentration of the proteins was measured using the BCA Protein Assay Kit (PC0020, Solarbio). Proteins (20 *μ*g) were separated by 12% sodium dodecyl sulfate-polyacrylamide gel electrophoresis and transferred onto polyvinylidene fluoride membranes (IPVH00010, Millipore). The membranes were blocked with 5% skim milk for 2 h at room temperature in Tris-buffered saline and incubated with primary antibodies against p-ERK1/2 (ab214036), JNK1/2/3 (ab208035), p-JNK1/2/3 (ab76572), and p-p38 (ab47363) from Abcam (UK), and ERK1/2 (MAB37123), p38 (PAB37381), AQP1 (PAB45863), and GAPDH (PAB36269) from Bioswamp (China), overnight at 4°C. GAPDH antibody (PAB36269, Bioswamp) was selected as an internal reference. All of the primary antibody dilution ratio is 1 : 1000. The membranes were then washed with Tris-buffered saline and incubated in goat anti-rabbit IgG secondary antibody (SAB43714, Bioswamp, 1 : 20000) for 2 h at room temperature. Immunoreactivity was visualized by the colorimetric reaction using Immobilon Western HRP (WBKLS0500, Millipore). The membranes were scanned with an Automatic Chemiluminescence Analyzer (Tanon 5200, Tanon).

### 2.9. Statistical Analyses

Statistical analyses were performed using SPSS 23.0 software. All data were presented as mean ± standard deviation (SD). Comparisons between the two groups were made using the independent-samples *t*-tests. The one-way ANOVA was used to compare differences among three or more groups, and the *post hoc* Fisher's least significant difference (LSD) test was used for the individual group comparisons. The values of *P* < 0.05 were considered statistically significant.

## 3. Results

### 3.1. Cirrhotic Ascites Lesions

As shown in Figure 1(a), the nucleus is stained with hematoxylin in a distinct blue color. The components in the cytoplasm and extracellular matrix were stained with eosin in different shades of red. The hepatocytes in the model group all showed steatosis, the pseudolobular structures were obvious in the fourth-week samples, and the sixth-week samples showed sclerotic necrotic features with disorganized hepatocyte arrangement, hepatocyte degeneration and necrosis, obvious proliferation of fibrous connective tissue, and extensive formation of pseudolobular structures. After ten weeks plus three days of carbon tetrachloride-olive oil injection, the rats in the model group increased their body weight slowly, and after the first week, a significant difference in body weight began to appear between the control group and the model group (*P* < 0.001), and the abdominal circumference coefficient (abdominal circumference/body weight) was calculated and found that the rats in the control group increased their abdominal circumference and body weight normally. On the contrary, the abdominal circumference of the model rats continued to increase with time. The increase in abdominal circumference was significantly greater in the model group than that in the control group at week 3 (Figure 1(b)). Thus, cirrhotic ascites can lead to an abnormal increase in abdominal girth and severe damage to the liver in rats.

### 3.2. QSZSP Alleviates Visceral Damage Caused by Cirrhotic Ascites

As shown in Figure 2, in the cirrhosis model group, the liver structure was disturbed and extensive vacuolar-like degeneration could be seen, and kidney tissue damage, glomerular hypertrophy, increase in the stroma of the thylakoid region, inflammatory cell infiltration, glomerular epithelial cell detachment, and the kidney tubules were dilated; peritoneal mesothelial cells were increased, the submesothelial stroma was thickened, and the peritoneal tissue was thickened. After four weeks of treatment with high-dose QSZSP, the liver tissue structure was basically intact, with centered nuclei and red-stained cytoplasm; most of the glomeruli had normal structure and normal tubules; peritoneal mesothelial cells were shed, and peritoneal tissue thickness was reduced compared with the model group.

### 3.3. QSZSP Regulates Liver Function-Related Factors in Rats with Cirrhotic Ascites

As shown in Figure 3, the concentrations of TBiL, AST, ALT, Cr, BUN, K, Na, and Ca in the model group were significantly higher (*P* < 0.001) than those in the control group and were significantly reduced after treatment with high doses of QSZSP. The concentrations of ALB in the model group were significantly lower (*P* < 0.001) than those in the control group, and their concentrations were significantly increased (*P* < 0.001) after treatment with a high dose of QSZSP. Combining the above two results, it can be found that QSZSP has the ability to modulate liver function-related factors to alleviate liver, kidney, and peritoneal damage caused by cirrhotic ascites.

### 3.4. QSZSP Regulates AQP1 Protein Expression in the Liver, Kidney, and Peritoneum

As shown in Figure 4, cirrhotic ascites leads to abnormally high expression of AQP1 protein in the liver, kidney, and peritoneum of rats (*P* < 0.001). Compared with the model group, AQP1 protein expression was reduced after treatment with a low dose of QSZSP and significantly reduced (*P* < 0.001) after treatment with a high dose of QSZSP, but AQP1 protein expression in the liver, kidney, and peritoneum was still higher than that in the control group at this time. QSZSP was able to inhibit AQP1 protein high expression caused by cirrhotic ascites.

### 3.5. QSZSP Inhibits the MAPK Signaling Pathway

As shown in Figure 5, the activation of p-ERK, p-JNK, and p-p38 in the model group was detected simultaneously in the liver, kidney, and peritoneum. The protein expression of p-ERK, p-JNK, and p-p38 was reduced after QSZSP treatment, and p-ERK, p-JNK, and p-p38 protein expression levels were significantly lower (*P* < 0.001) after a high-dose QSZSP treatment than those in the model group.

### 3.6. QSZSP Induces Abdomen Circumference in Rats with Cirrhotic Ascites

As shown in Figure 6, after four weeks of treatment, the model group's rat body weight is always lower than the other three groups, and after treatment with QSZSP at high dose, rats with cirrhotic ascites showed a significant increase in body weight, and the body weight of rats in the QSZSP low-dose treatment group was also higher than that of the model group (Figure 6(a)). Interestingly, the rats in the QSZSP high-dose group showed a decreasing trend in abdominal circumference along with an increase in body weight, and after four weeks of treatment, the rats in the QSZSP high-dose group were significantly lower than the model group. Combined with the results of HE staining, it could indicate that QSZSP alleviated the organ damage caused by cirrhotic ascites and reduced the abnormal growth of abdominal circumference.

## 4. Discussion

Cirrhosis ascites is a pathological phenomenon of fluid accumulation in the abdominal cavity caused by a combination of factors during the decompensated phase of cirrhosis and is the most common first event in the decompensated phase of cirrhosis. It not only brings unbearable pain to patients with liver disease and significantly reduces the quality of life, but also causes water-electrolyte disorders and deterioration of the body's internal environment, which can lead to serious complications such as liver encephalopathy, upper gastrointestinal bleeding, and hepatorenal syndrome, and is one of the main factors leading to death in patients with liver disease [31, 32]. Studies have shown that patients with cirrhotic ascites have a 3-year morbidity and mortality rate of 50% and a 5-year survival rate of only 5–10% [33]. This study not only found that cirrhotic ascites led to severe liver, peritoneum, and kidney damage, but also found that rats with cirrhotic ascites had slowed weight gain and excessive growth in abdominal circumference (Figure 1). After 4 weeks of treatment, the rats began to gain weight and their abdominal circumference was reduced (Figure 6).

Tie et al. [29] found that in prostate cancer cells, hypoxia induced AQP1 protein upregulation in a p38-dependent manner and that AQP1 was induced by hypoxia at the transcriptional level and that AQP1 regulation in PC-3M was dependent on calcium, PKC, and p38MAPK as well as oxygen tension. AQP1 is widely expressed in lymphatic vessels, capillaries, and endothelial cells of small veins and is distributed in the liver, peritoneum, kidney, pleura, respiratory tract, digestive tract from esophagus to colon, cardiac muscle, smooth muscle, and brain [24]. Huebert et al. [34] found that in the early stages of liver fibrosis, AQP1 expression on liver tissue cell membranes increased accordingly as the degree of liver fibrosis progressed. Liu et al. [30, 35] found that peptidoglycan is an inhibitor of the p38 MAPK transduction pathway and lipopolysaccharide is an inhibitor of the p38/JNK/ERK pathway ultimately acting on the AQP1 gene causing downregulation of AQP1 expression in human pleural mesothelial cells and that the reduction in AQP1 expression is dose-dependent and time-dependent. In this study, QSZSP was able to inhibit AQP1 protein high expression caused by cirrhotic ascites in the “liver-peritoneum-kidney” axis of cirrhotic ascites rats. QSZSP was able to inhibit AQP1 protein high expression caused by cirrhotic ascites, and the MAPK signaling pathway in the “liver-peritoneum-kidney” axis was also inhibited at this time. This demonstrated that the activation of MAPK signaling pathway was involved in organ damage in the “liver-peritoneum-kidney” axis of cirrhotic ascites rats and was associated with AQP1. Finally, it was found that the treated rats had lower Cr and TBiL and significantly higher ALB in serum, which, combined with the increase in body weight after treatment, indicated that QSZSP had some effect on improving the quality of life.

However, for the treatment of patients with cirrhotic ascites, medicine will obviously increase water intake, which contradicts the principle of water restriction in this disease; in particular, for patients with a large amount of ascites, medicine administration will further increase the patient's abdominal distension symptoms, and their compliance is poor. Chinese medicine is an important external treatment method in TCM, which can solve the contradiction between traditional Chinese medicine and the treatment of cirrhotic ascites with water restriction and can act directly on the diseased area. The development of the formulation process, quality standard, and safety of the gel form of QSZSP has been completed in the previous phase [36–39].

Previous studies on the mechanism of ascites formation in cirrhosis have mainly focused on the pathological role of the liver and kidney, such as the alteration of portal hemodynamics by cirrhosis, the water and sodium retention effect of the kidney, or the hormonal changes triggered by both, neglecting the role of the peritoneum and the role of the liver-peritoneum-kidney as an organic whole in the formation of ascites in cirrhosis.

Based on the previous study, this study took the pathological nature of water metabolism disorder in cirrhotic ascites as the starting point and was the first to propose the hypothesis that the “liver-peritoneum-kidney” axis is a functional axis of water metabolism that is involved in the “production-absorption-exhaustion” of peritoneal fluid with aquaporins protein as the common material basis and plays a key role in the formation of cirrhotic ascites. It was proved that QSZSP can inhibit the activation of MAPK signaling pathway and protect liver function in cirrhotic ascites rats, and it was found that AQP1 of “liver-peritoneal-kidney” axis plays a facilitating role in the process of ascites in cirrhosis ascites. The study also demonstrated that QSZSP regulates AQP1 expression in the “liver-peritoneal-kidney” axis, thus achieving the therapeutic effect of blocking ascites. It is clear that QSZSP inhibits AQP1 expression in the liver, peritoneum, and kidney, thus reducing abdominal girth. This process is related to the inhibition of MAPK pathway activation by QSZSP.

Many studies have found that the MAPK signaling pathway is involved in the regulation of ascites in cirrhosis. In this study, we found that the activation of MAPK signaling pathway was inhibited after QSZSP treatment, but whether QSZSP targets the MAPK signaling pathway for the treatment of cirrhotic ascites is unknown in this study. As a limitation of this study, perhaps the targeting relationship of MAPK signaling pathway in QSZSP for the treatment of cirrhotic ascites will be verified *in vitro* in future studies of liver.

## 5. Conclusion

QSZSP inhibits MAPK activation and AQP1 protein expression in the “liver-peritoneal-kidney” axis to alleviate ascites injury in cirrhosis.

## Figures and Tables

**Figure 1:** Cirrhotic ascites lesions. (a) HE staining of liver tissue at the fourteenth week (×100). (b) Abdominal circumference index (abdominal circumference/body weight) during modeling. (c) Body weight during modeling. Scale bar = 50 *μ*m.  ^*∗∗∗*^*P* < 0.001 Con vs. Mod.

**Figure 2:** Tissues of liver, kidney, and peritoneum HE staining (×100). Scale bar = 50 *μ*m.

**Figure 3:** Concentrations of TBiL, AST, ALT, Cr, BUN, K, Na, Ca, and ALB in different treatment groups.

**Figure 4:** QSZSP inhibits AQP1 protein expression in the liver, kidney, and peritoneum of cirrhotic ascites. (a) Expression of AQP1 protein in IHC staining (×100). Scale bar = 50 *μ*m. (b) IOD of AQP1 in the liver. (c) IOD of AQP1 in the kidney. (d) IOD of AQP1 in the peritoneum. (e) Expression of AQP1 protein in Western blot. (f–h) Relative expression of AQP1 protein in the liver, peritoneum, and kidney, and GAPDH is loading control.  ^*∗∗*^*P* < 0.01 vs. Con,  ^*∗∗∗*^*P* < 0.001 vs. Con, ^##^*P* < 0.01 vs. Mod, ^###^*P* < 0.001 vs. Mod.

**Figure 5:** QSZSP inhibits the MAPK signaling pathway. (a, d) Expression of p-ERK1/2, p-JNK1/2/3, and p-p38 protein in the liver. (b, e) Expression of p-ERK1/2, p-JNK1/2/3, and p-p38 protein in the peritoneum. (c, f) Expression of p-ERK1/2, p-JNK1/2/3, and p-p38 protein in the kidney.  ^*∗∗∗*^*P* < 0.001 vs. Con, ^###^*P* < 0.001 vs. Mod. *Note.* 1: control group, 2: model group, 3: QSZSP low-dose group, and 4: QSZSP high-dose group.

**Figure 6:** QSZSP induces abdomen circumference in rats with cirrhotic ascites. (a) The body weight of QSZSP after four weeks of treatment. (b) Abdominal circumference index (abdominal circumference/body weight) of QSZSP after four weeks of treatment.  ^*∗∗∗*^*P* < 0.001 Con vs. Mod.

**Table 1:** The changes in body weight (g) during 15 weeks.

Time (week)	Con	Mod	QSZSP low dose	QSZSP high dose
2	240.62 ± 8.76	231.97 ± 7.16	239.07 ± 8.88	241.32 ± 6.00
2.5	274.57 ± 13.79	244.28 ± 10.14	242.30 ± 14.88	246.90 ± 9.78
3	306.48 ± 11.66	240.08 ± 10.87	253.33 ± 20.08	250.90 ± 17.92
3.5	337.52 ± 13.11	244.98 ± 10.41	264.48 ± 14.18	252.92 ± 16.52
4	373.97 ± 13.15	246.87 ± 15.24	269.18 ± 22.74	262.25 ± 24.54
4.5	408.90 ± 14.12	259.20 ± 13.81	272.98 ± 14.06	262.88 ± 28.43
5	406.57 ± 14.39	263.95 ± 14.27	275.33 ± 15.39	265.90 ± 30.20
5.5	411.27 ± 18.97	266.62 ± 19.88	283.02 ± 14.66	269.65 ± 32.02
6	418.87 ± 19.39	267.30 ± 26.75	278.12 ± 19.41	265.18 ± 33.80
6.5	420.77 ± 23.51	270.97 ± 29.79	281.47 ± 18.66	267.65 ± 33.37
7	438.87 ± 24.75	266.90 ± 26.26	284.62 ± 22.64	269.08 ± 36.85
7.5	445.37 ± 30.10	275.10 ± 21.13	288.15 ± 20.96	271.12 ± 35.28
8	456.02 ± 34.16	279.10 ± 19.79	289.05 ± 14.94	267.52 ± 29.48
8.5	461.45 ± 39.24	277.60 ± 21.83	292.28 ± 17.86	272.82 ± 27.29
9	474.13 ± 43.54	282.35 ± 24.55	294.52 ± 20.95	270.83 ± 30.05
9.5	476.95 ± 45.68	285.43 ± 25.48	293.98 ± 17.88	273.87 ± 23.30
10	482.80 ± 38.05	283.07 ± 25.10	289.20 ± 19.57	273.80 ± 25.58
10.5	498.40 ± 37.98	279.98 ± 24.91	283.63 ± 27.88	268.77 ± 22.97
11	500.08 ± 34.11	276.07 ± 26.91	273.55 ± 27.04	273.88 ± 27.42
11.5	515.92 ± 40.80	275.50 ± 22.32	272.35 ± 33.01	276.53 ± 32.26
12	524.85 ± 38.18	274.00 ± 26.76	276.17 ± 27.98	272.23 ± 32.27
12.5	537.27 ± 36.80	271.18 ± 28.56	270.63 ± 25.96	272.13 ± 28.11
13	566.72 ± 37.67	284.08 ± 30.70	282.43 ± 29.67	301.62 ± 23.60
14	583.90 ± 34.03	296.22 ± 33.35	294.28 ± 33.14	329.77 ± 27.03
15	612.17 ± 41.29	332.53 ± 18.22	339.03 ± 10.94	394.83 ± 13.66
16	632.90 ± 42.57	341.47 ± 15.02	362.20 ± 9.71	427.40 ± 11.89

Data presented as mean ± standard deviation.

**Table 2:** The changes in abdominal circumference (mm) during 15 weeks.

Time(week)	Con	Mod	QSZSP low dose	QSZSP high dose
2	86.82 ± 10.10	83.42 ± 6.08	83.97 ± 2.57	88.95 ± 5.24
2.5	97.93 ± 8.89	91.67 ± 7.76	91.50 ± 3.84	88.97 ± 7.59
3	107.78 ± 7.12	84.52 ± 8.14	92.47 ± 8.92	91.57 ± 9.15
3.5	116.95 ± 8.95	92.30 ± 7.04	94.78 ± 7.58	93.72 ± 9.83
4	130.27 ± 8.90	97.50 ± 7.68	104.23 ± 6.31	98.73 ± 9.81
4.5	150.05 ± 12.11	100.03 ± 7.61	106.33 ± 4.13	103.20 ± 15.95
5	144.35 ± 14.13	108.78 ± 10.27	110.85 ± 7.32	108.58 ± 15.77
5.5	142.02 ± 11.11	110.63 ± 10.71	115.10 ± 8.89	111.40 ± 17.23
6	157.02 ± 9.70	109.18 ± 9.64	119.68 ± 10.69	115.10 ± 14.29
6.5	154.47 ± 13.95	116.42 ± 14.45	116.17 ± 8.02	112.65 ± 13.56
7	149.68 ± 8.13	114.72 ± 16.26	120.90 ± 11.55	114.57 ± 20.11
7.5	165.20 ± 12.73	124.82 ± 16.89	123.07 ± 12.84	118.77 ± 16.80
8	171.13 ± 7.42	125.50 ± 14.24	123.18 ± 9.90	120.28 ± 13.06
8.5	168.32 ± 22.96	136.28 ± 13.62	141.88 ± 11.82	124.18 ± 14.54
9	166.77 ± 25.63	137.53 ± 11.23	139.52 ± 6.78	128.63 ± 15.32
9.5	175.60 ± 19.28	137.00 ± 9.18	145.05 ± 6.80	127.73 ± 16.29
10	162.43 ± 13.10	140.27 ± 17.08	142.58 ± 9.35	134.80 ± 15.86
10.5	167.73 ± 12.37	143.18 ± 17.91	137.97 ± 15.70	132.43 ± 11.86
11	170.40 ± 17.75	133.67 ± 16.74	129.23 ± 13.34	135.38 ± 8.86
11.5	174.67 ± 16.79	131.15 ± 12.09	139.08 ± 15.77	130.03 ± 21.11
12	176.17 ± 18.18	131.75 ± 20.23	142.13 ± 18.74	137.10 ± 17.83
12.5	183.68 ± 16.49	132.83 ± 11.32	130.85 ± 19.06	135.52 ± 15.62
13	190.35 ± 20.90	155.17 ± 17.92	153.37 ± 12.49	149.97 ± 14.59
14	192.75 ± 16.63	170.27 ± 20.43	164.73 ± 11.44	161.17 ± 16.53
15	211.00 ± 14.26	198.93 ± 6.09	181.20 ± 8.63	177.73 ± 18.77
16	214.10 ± 17.34	213.80 ± 3.89	189.43 ± 7.17	185.03 ± 17.42

Data presented as mean ± standard deviation.

## Data Availability

The data used to support the findings of this study are available from the corresponding author upon request.

## Additional Points

(i) Qi Sui Zhu Shui plaster inhibits MAPK activation in cirrhotic ascites rat. (ii) Qi Sui Zhu Shui plaster suppressed cirrhotic ascites-induced liver-peritoneum-kidney damage *in vivo*. (iii) Qi Sui Zhu Shui reduced abdominal circumference thickness by inhibiting the overexpression of AQP1.
